The article "The impact of environmental information disclosure quality on green innovation of high-polluting enterprises" was retracted in 2025. Reasons: an official misconduct investigation; compromised peer review; a compromised editor; unreliable results or conclusions.

# The impact of environmental information disclosure quality on green innovation of high-polluting enterprises

**DOI:** 10.3389/fpsyg.2022.1069354

**Published:** 2022-12-13

**Authors:** Lizhao Du, Xinpu Wang, Jie Peng, Gaoyang Jiang, Suhao Deng

**Affiliations:** ^1^School of Economics and Management, Lanzhou Jiaotong University, Lanzhou, China; ^2^Jiangsu Institute of Industrial Development Research, Nanjing University of Finance and Economics, Nanjing, China; ^3^Institute of Food and Strategic Reserves, Nanjing University of Finance and Economics, Nanjing, China

**Keywords:** environmental disclosure quality, green innovation, financing constraints, cash reserves, high-polluting enterprises

## Abstract

With the gradual increase of social awareness of environmental protection, environmental information disclosure has become the key for enterprises to accept social supervision and fulfill their social responsibility. This study examines the high-polluting enterprises that were listed on Chinese A-shares between 2008 and 2021. The influence of environmental information disclosure quality on green innovation is examined using ordinary least squares (OLS) as a benchmark model. The results show that the improvement of environmental information disclosure quality of high-polluting enterprises can significantly improve the quantity and quality of green innovation of enterprises and are mediated by alleviating financing constraints and enhancing cash reserves. Moreover, improving the quality of environmental information disclosure of highly polluting enterprises has a more significant contribution to the quantity and quality of green patents of non-state-owned enterprises, enterprises located in central and eastern China, and large enterprises. The findings of this paper provide theoretical support for achieving a “win-win” situation of environmental protection and green innovation.

## Introduction

After the subprime crisis, most countries are facing the double test of economic recession and environmental degradation and most nations are currently experiencing a double difficulty of economic contraction and environmental damage following the subprime crisis. Therefore, it has become a top priority for governments and international organizations to concentrate on increasing energy use efficiency, decreasing resource consumption, and implementing an environmentally friendly green development model while sustaining economic growth. China’s economy has grown rapidly for almost 40 years thanks to reform and opening up, but these changes have also brought about significant ecological and environmental pollution issues. Economic and social development in China is being severely hampered by severe resource and environmental limits brought on by the primitive economic development model of high input and high emission (Han et al., 2022; Yuan and Cao, 2022). In order for China to achieve high-quality economic development, it is now essential to shift from resource-driven, sloppy development to innovation-driven, green development. China first prioritized innovation in 2015 and stressed the significance of green development, calling for a green transformation of the development method and fostering high-quality economic development and high-level ecological conservation. This demonstrates that promoting a “win-win” situation for China’s economic growth and environmental protection depends heavily on green innovation (Cao et al., 2021).

Green innovation is typically thought of as a notion that is closely tied to green technology and green technology innovation. It is based on green technology innovation and includes initiatives for institutional and organizational structure innovation related to green technology (Hur et al., 2013; Arenhardt et al., 2015; Cao et al., 2022). In contrast to conventional innovation activities, green innovation places a focus on the adoption of innovative technological concepts to achieve efficient energy use and considerable reductions in pollutant emissions while receiving matching economic benefits (Chen and Hung, 2014), that is, the goal of green innovation is to obtain positive environmental advantages in addition to reducing environmental pressure (Driessen et al., 2013; Yang et al., 2021b). Therefore, green innovation is an essential tool for enterprises to achieve economic development and environmental protection (Fernando et al., 2019). The existing literature on green innovation primarily focuses on the impact that green innovation has and the drivers of green innovation. First, the influence of green innovation on other factors. According to some academics, increasing the degree of green innovation can successfully improve the energy consumption structure of businesses (Jiang et al., 2020; Yang et al., 2021a), raise energy utilization efficiency (Sun et al., 2019; Yang et al., 2022), and decrease the intensity of pollutant emissions (Dong et al., 2022; Yi et al., 2022; Ren et al., 2022b), and the intensity of pollutant emissions, all of which will raise people’s quality of life (Aguilera-Caracuel and Ortiz-de-Mandojana, 2013; Amore et al., 2015; Burlea-Schiopoiu et al., 2022). Additionally, businesses that invest in green innovation can boost their financial performance (Rezende et al., 2019; Xie et al., 2022), environmental performance (Singh et al., 2020), and competitive advantages (Barforoush et al., 2021). Second, internal corporate drives and external environmental forces have been examined when examining the drivers of green innovation. From the perspective of external environmental forces, in order to promote enterprises to adopt more proactive environmental strategies to cope with the environmental challenges they face, the government has implemented several environmental regulatory systems to encourage the green transformation of enterprises’ production activities, such as the emissions trading system and the development of environmental subsidies (Hsu et al., 2011). By increasing their emissions costs and level of green innovation, the emissions trading system can “push” companies to invent environmentally friendly processes to lessen their reliance on antiquated, polluting manufacturing techniques (Porter and Linde, 1995). On the other hand, government subsidies offer a source of funding for businesses to implement green innovation, alleviate the lack of resources businesses face to carry out green innovation, and lower the cost of green innovation for businesses (Montmartin and Herrera, 2015), allay managers’ worries about the unpredictability of innovation activities, and thereby increase businesses’ ex-ante tolerance for green innovation risks (Stiglitz, 2015). From the internal corporate drives, to ensure their social legitimacy and gain a good social reputation, enterprises will choose to implement green innovation strategies and establish a green corporate image (Liu, 2022), so that enterprises can gain certain competitive advantages (Arenhardt et al., 2015; Albort-Morant et al., 2018), win the trust of their suppliers and customers (Haddoud et al., 2021), differentiate their products from those of their rivals, reduce environmental pollution, improve their environmental performance, and lower environmental costs in the production process in general (Küçükoğlu and Pınar, 2015; Singh et al., 2020; Dong et al., 2022; Yi et al., 2022), as well as stimulate new market demand.

Green innovation, however, comes with significant risks and demands significant R&D investment from businesses. Entrepreneurs usually lack the motivation to engage in independent R&D. Thus, governments introduce various environmental regulation laws to encourage businesses to engage in green innovation (Feng and Chen, 2018; Zhang et al., 2019; Meng et al., 2020), one of which is the environmental information disclosure (EID). EID is a set of actions taken by businesses to disclose their environmental performance, environmental points publicly, and environmental protection inputs in their business operations through official corporate websites, social responsibility reports, and corporate annual reports (Kreuze et al., 1997; Jiao et al., 2017; Schiopoiu Burlea, 2019; Ding et al., 2022), and it serves as a critical barometer for assessing how seriously businesses take their social responsibility. The current study on EID is divided into the following two main areas: the factors that influence the quality of EID. From the perspective of external pressure, the media can promote public awareness of corporate governance concerns and improve the quality of corporate EID from the standpoint of external pressure because it is a crucial weapon for influencing public opinion (Fan et al., 2020). Additionally, institutional pressure from various governmental environmental regulatory instruments enhances the standard of EID by businesses (Ren et al., 2020). Regarding internal aspects, rationalizing corporate governance can considerably enhance the quality of a company’s EID (Raimo et al., 2021). Moreover, executive traits and the type of a company’s property rights can also impact the disclosure’s quality (Wang et al., 2020; Zhang et al., 2021). The second is the impact of EID. Improving the quality of EID can effectively enhance corporate value and corporate performance (Li et al., 2017; Wang et al., 2020), reduce corporate risk (Chang et al., 2021), and alleviate the financing constraints faced by companies (Li Q. et al., 2022), but the effect on a company’s profitability is questionable (Yin et al., 2019; Pedron et al., 2021). The literature has also looked at the connection between EID and green innovation, mainly as a quasi-natural experiment to look into the effects of installing an EID system on green innovation at the city level (Li G. et al., 2022; Zhang S. et al., 2022). Little literature has explored the relationship between the quality of EID and corporate green innovation from the perspective of firms. So, can increasing the quality of EID increase the amount of green innovation in high-polluting enterprises? What mechanisms does this advertising effect travel through? Are the impacts heterogeneous? To fill this gap, this paper examines the relationship between corporate green innovation and the quality of EID of high-polluting enterprises, using high-polluting enterprises listed on Chinese A-shares from 2008 to 2021 as a research sample. The environmental activities and behaviors of high-polluting enterprises are more sensitive to environmental regulation-type policies. They are a source of significant pollutant emissions, making it necessary and practical to investigate the impact of EID on the green innovation of high-polluting enterprises.

Specifically, this paper calculates the EID quality of high-polluting enterprises listed in Chinese A-shares from 2008 to 2021. It examines the impact of EID quality on corporate green innovation from two perspectives: the quantity and quality of green patent applications explore the transmission path of this impact, and discusses the heterogeneity of this impact from three perspectives: the ownership structure of the firm, the location of the firm, and the size of the firm.

The marginal contributions of this paper compared to previous studies are as follows: First, this paper analyzes the factors affecting corporate green innovation from the perspective of environmental information disclosure quality. The existing literature mostly takes the ‘Guidelines on Environmental Information Disclosure for Listed Companies’ issued by Shanghai Stock Exchange in 2008 as a quasi-natural experiment to study the impact of mandatory environmental information disclosure on corporate innovation, and little literature has explored the relationship between environmental information disclosure quality and corporate innovation (Ren et al., 2020). This paper explores the impact of different types of environmental information disclosure on the quantity and quality of firms’ green innovation from the perspective of environmental information disclosure quality, which enriches the research perspective of influencing firms’ green innovation. Secondly, the text explores how the improvement of the quality of environmental information disclosure can motivate enterprises to engage in green innovation through the internal enterprise. The existing literature mostly explores the impact of environmental information disclosure on enterprises from the perspective of external pressure, such as the media attention faced by enterprises and the relationship between enterprises and the government (Fan et al., 2020; Cailou et al., 2021). This paper explores whether the improvement of environmental information quality can be achieved by alleviating the financing constraints faced by enterprises from the internal enterprise and improving their cash flow reserves. Third, this paper provides theoretical support and empirical evidence for policymakers and relevant enterprises to further understand the importance of improving the quality of environmental information disclosure by studying the impact of environmental information disclosure quality on corporate green innovation.

The remainder of the paper is structured as follows: Section II presents the theoretical analysis and research hypotheses, and Section III describes the research design, including data sources, variable definitions, and model settings. Section IV presents the results and discussion of the empirical evidence, and section V presents the conclusion.

## Theoretical analysis and research hypothesis

Government and public concern about business environmental performance is growing as society becomes more environmentally conscious. This institutional and social pressure is forcing companies to improve the quality of their EID to alter stakeholders’ perceptions of their environmental performance and thereby enhance their social standing (Merkl-Davies et al., 2011; Meng et al., 2013; Li et al., 2018). According to the legitimacy organization theory, in order for an enterprise to continue to exist and operate over the long term, it must adhere to the relevant policy standards and public social expectations, and its production and operation activities must comply with various institutional norms, which implies that the enterprise must take on the relevant social responsibility (Patten, 1992; Hooghiemstra, 2000; Cho and Patten, 2007; Mohamad Nur et al., 2020). Society is particularly concerned about its environmental performance because it is an environmentally sensitive business. A high-polluting enterprise must present a positive public image of being brave enough to take on social responsibility to demonstrate its environmental legality. To do this, the company must disclose environmental information that complies with social expectations and policy requirements, meaning that it is under internal and external pressure to improve the quality of its EID (Tinker et al., 1982, 1991). A systematic study of EID of all Lithuanian enterprises found that compared to other industries, energy, steel, and building materials, which have a more significant impact on the environment, are more inclined to disclose higher quality environmental information to the community (Leitoniene and Sapkauskiene, 2015). In addition to stating their environmental protection philosophies and other qualitative information, high-quality EID mandates that enterprises disclose their environmental management performance, environmental protection investment, and other quantitative information. Additionally, it mandates that enterprises continuously improve their energy consumption structure, energy use efficiency, resource use efficiency, and pollutant control. In other words, businesses must continually boost their R&D spending on environmental protection initiatives and strengthen their capacity for green innovation to guarantee the consistent development of their environmental performance and forge a green corporate identity. Based on the above analysis, the following hypotheses are proposed in this paper.

*H1*: EID can promote green innovation in high-polluting enterprises.

High-quality EID can show the public that businesses are brave in upholding their social obligations, enhance investors’ perceptions of businesses overall, ease the financial challenges businesses face (Clarkson et al., 2013; Liu et al., 2020; Wang et al., 2021; Zhang B. et al., 2022), and provide funding for businesses to launch green innovation projects. Finance-related limitations significantly impact the R&D innovation activities of businesses, characterized by high adjustment costs and high unpredictability, and are less eager to launch innovation initiatives when they are more severe. Using Spanish firms from 2005 to 2013, García-Quevedo et al. (2018) found that financing constraints significantly constrain the establishment of innovation projects at the conception stage of the innovation project; Ghisetti et al. (2015), on the other hand, examines the impact of financing constraints on green innovation in EU SMEs and finds that financing constraints significantly hinder EU SMEs from engaging in green innovation. According to information asymmetry and principal-agent theory, agents may, out of self-interest, give their principals with inaccurate and incomplete information, which could influence the way investors make decisions (Cho and Patten, 2007; Delmas and Toffel, 2008; Ciliberti et al., 2011; Cao et al., 2013). High-polluting businesses must disclose their environmental information to investors in order to demonstrate their courage in accepting social responsibility and to address the issue of environmental information asymmetry between investors and businesses. From the perspective of investors, high-polluting businesses have more serious environmental risks than other types of businesses. As a result, to minimize the issue of adverse selection, investors will inevitably gravitate toward businesses that provide better EID, increasing the likelihood that their loans will be repaid in the future. High-quality EID can effectively ease the financial challenges faced by high-polluting enterprises in the process of R&D and innovation, signal to investors that companies are actively fulfilling their environmental obligations, and assist investors in identifying socially responsible companies. Du (2018) investigates the effect of EID on the financing constraints of Chinese A-share listed companies and finds that EID can effectively alleviate information asymmetry between domestic and foreign investors, thereby reducing foreign share price discounts and helping firms attract overseas financing. Based on the above analysis, this paper proposes the following hypothesis.

*H2*: EID promotes green innovation in high-polluting enterprises by alleviating financing constraints.

Enhancing an organization’s EID capabilities also increases its visibility, fosters a green and environmentally conscious corporate image, boosts operating income, and provides the financial stability necessary for it to continue to fund new projects. According to the stakeholder theory, businesses must also consider their external stakeholders, such as the government and society, in addition to their internal stakeholders, such as directors and managers (Brammer et al., 2007; Delmas and Toffel, 2008; Aguinis and Glavas, 2012; Khan et al., 2013). Companies must fulfill external stakeholders’ expectations for corporate social responsibility in order to develop their relationships with them and obtain a corresponding competitive advantage as the public’s concern about environmental issues grows. Disclosure of high-quality environmental information benefits businesses in several ways, including market scale expansion, product development to suit consumer demand, customer retention, profitability improvement, and cash flow growth (Kassinis and Soteriou, 2003; Hart and Dowell, 2011). Chopra and Wu (2016) studied the impact of environmental performance on the operating performance of companies in the computer and electronics industry in the United States from 2000 to 2011. They found that improvements in environmental performance significantly contributed to companies increasing their operating income. An innovation project requires a significant amount of capital investment from the beginning to the end, and if the capital chain breaks in the middle of the process, the project cannot be implemented smoothly. In contrast, cash flow, an uncommitted and unabsorbed financial resource with almost no significant reallocation and deployment, gives companies more discretion to quickly replace the missing part of resources in the R&D process and meet their investment needs (Tabesh et al., 2019). Hall (1992) used a sample of public trade manufacturing firms from 1973 to 1987 as a study. A significant positive relationship between a firm’s cash flow and its investment in innovation was found using a dynamic gas pedal model. With a sample of U.S. manufacturing firms from 1970 to 2006, Brown and Petersen (2011) analyze the impact of cash holdings on firms’ investment in R&D and find that firms with higher constraints on financing can smooth their R&D expenditures through liquidity reserves. Based on this, this paper proposes the following hypothesis.

*H3*: EID promotes green innovation in high-polluting enterprises by enhancing firms' cash reserves.

## Research design

### Sample and data

Using the 2008–2021 Chinese A-share listed enterprises as the original sample, we filtered the listed enterprises belonging to high-pollution industries according to the ‘Guide to Environmental Information Disclosure of Listed Companies (Draft for Comment)’ issued by the Ministry of Environmental Protection and the ‘Industry Classification Guidelines for Listed Companies’ revised by the China Securities Regulatory Commission in 2012^1^, and excluded the enterprises that had been delisted during the sample period, the enterprises with some missing data and the enterprises with negative book value of owner’s equity. In order to control the influence of extreme values, all continuous variables are subjected to an upper and lower 1% tailing process, and finally 6,986 observations are obtained, among which 499 are high-polluting enterprises. The number of patent applications in this paper was obtained from the patent application data (2008–2021) of A-share listed companies provided by China Research Data Service Platform (CNRDS), and then the green patents applied by listed companies were screened according to the “Green List of International Patent Classification” issued by the World Intellectual Property Organization (WIPO) in 2010. The number of green patent applications of high-polluting enterprises from 2008 to 2021 was finally obtained by filtering. The remaining corporate-level data, such as environmental information disclosure, number of board of directors, number of independent directors, highest shareholder ownership, net income, year-end fixed assets, total debt, time of establishment, and earnings per share, were obtained from China Stock Market & Accounting Research (CSMAR; 2008–2021).

### Model setting

To test the impact of high-polluting enterprises on the quality of EID on green innovation, the benchmark regression was estimated using ordinary least squares (OLS) and was set as follows:


(1) $${\mathrm{lnGInno}}_{\mathrm{it}}=\beta_{0}+\beta_{1}{\mathrm{lnEID}}_{\mathrm{it}}+\beta_{2}X_{\mathrm{it}}+\mu_{j}+\sigma_{t}+\varepsilon_{\mathrm{it}}$$

where i represents the firm; t represents time; j represents industry; ${\mathrm{lnGInno}}_{\mathrm{it}}$ is the natural logarithm of the firm’s green patent applications, and ${\mathrm{lnEID}}_{\mathrm{it}}$ is the natural logarithm of the firm’s environmental disclosure quality; $X_{\mathrm{it}}$ represents a series of control variables, including the number of board of directors (Bsize), the proportion of independent directors (Bratio), the highest shareholding ratio (Sratio), the firm’s growth prospect (Future), firm size (lnAsset), firm debt (Lev), firm maturity (Age), and firm profitability (Share); $\mu_{j}$ is an industry fixed effect; $\sigma_{t}$ is a time fixed effect; and $\varepsilon_{\mathrm{it}}$ is a random error term.

### Definition of main variable

#### Explained variable: Green innovation (GInno)

The key reasons for utilizing the quantity of green patent applications to gauge an organization’s level of green innovation are as follows: first, the quantity of green patents allows for a more precise assessment of an organization’s level of green innovation output. The established literature typically uses enterprise R&D investment or innovation subsidies to measure enterprises’ innovation level, but it can be challenging to distinguish between R&D costs or innovation subsidies invested by enterprises in the field of green technology. This paper uses the index list of environment-friendly international patent classification released by the World Intellectual Property Organization (WIPO) in 2010 to identify the green patents of enterprises. Secondly, the number of patent applications is more timely and reliable. Studies show that patents have an impact on the production activities of enterprises at the time of application (Jiang et al., 2020), while Chinese patents take a long time from application to approval and authorization, with invention-type patents usually taking 1–2 years to be granted, and patent authorization may also be interfered by the rent-seeking behavior of patent administration departments. Therefore, this paper identifies and accounts for the green patent data of high-polluting enterprises in China from 2008 to 2021 using the WIPO’s index list of environment-friendly international patent classifications. It then uses the natural logarithm of the total number of green patent applications plus one as an indicator of enterprises’ green innovation activities (lnGInno), where the higher the value, the more green innovation is being done. Additionally, since invention-type patents have a higher technical content than utility models, the proportion of green invention patent applications to all green patent applications is calculated in this paper. The natural logarithm is then taken after adding 1 to test the impact of high-polluting enterprises’ EID on the quality of those enterprises’ green patent applications(lnGInnoQ).

#### Explanatory variable: Quality of EID (EID)

There are two main approaches to measuring the quality of EID in the existing literature: one is to directly use the results of assessments of corporate EID published by organizations such as Hexun.com, R&L Global, and Blue Book. Another is to construct an EID index to measure the quality of companies’ EID by referring to the ‘sustainability reporting guidelines issued by the Global Reporting Initiative (GRI) and the content related to EID issued by the ‘EID Scheme (Trial)’ issued by the Chinese Ministry of Environmental Protection. With reference to the existing literature (Fan et al., 2020; Wang et al., 2020), the environmental data disclosed by companies are classified into soft indicators (EIDS) and complex indicators (EIDH) according to the concept of Boesso and Kumar (2007). Soft indicators include qualitative data like environmental protection philosophy and environmental goals, while complex indicators include quantitative data like pollutant emissions, pollutant management, and green innovation investment (Table 1). Disclosure is given a value of 1, else 0, for soft indicators. Nondisclosure is given a value of 0, qualitative description is given a value of 1, and quantitative description is given a value of 2, all for complex indications. To acquire the quality of the EID of firms, the soft and hard indicators are finally included (Eq. 2), and the natural logarithm is also taken into account to control any potential heteroskedasticity.


(2) $$\begin{array}{c} \left\{\begin{array}{c} EID_{it}=EIDS_{it}+EIDH_{it}\\ EIDS_{it}=\overset{n}{\underset{j=1}{\sum }}EIDS_{ijt};j=1,2,\ldots ,10\\ EIDH_{it}=\overset{m}{\underset{j=1}{\sum }}EIDS_{ijt};j=1,2,\ldots ,17 \end{array}\right. \end{array}$$

**Table 1:** EID quality index system.

Indicator properties	Disclosure information	Specific category	Assignment method
Soft	Environmental Management	Environmental protection concept, environmental protection objectives, environmental management system, environmental protection education and training, environmental protection special action, environmental events emergency mechanism, environmental protection honors or awards, “three simultaneous” system	Disclosure is 1 Otherwise 0
	Environmental Regulation and Certification	ISO14001 certification or not, ISO9001 certification or not	Pass is 1 Otherwise 0
Hard	Environmental liabilities	Wastewater emissions, COD emissions, SO_2_ emissions, CO_2_ emissions, soot and dust emissions, industrial solid waste generation	Non-disclosure is 0 Qualitative disclosure is 1 Quantitative disclosure is 2
	Environmental Performance and Governance	Emission reduction treatment of exhaust gas, wastewater emission reduction treatment, dust, smoke and dust treatment, solid waste utilization and disposal, noise, light pollution, radiation and other governance, clean production implementation	
	Environmental Investment	Project name, input cost	

#### Mediator variable

##### Financing constraints (SA)

The representative methods of enterprise financing constraints are KZ index (Lamont et al., 2001), WW index (Whited and Wu, 2003), and SA index (Hadlock and Pierce, 2010). In contrast to KZ index and WW index, which classify the types of financing limitations of firms based on their financial reports, SA index produces SA index utilizing enterprise size and enterprise age, successfully avoiding endogeneity interference. As a result, this paper chooses the SA index to measure the financing constraints on high-polluting enterprises, which is calculated as:


(3) $$\begin{array}{c} {\mathrm{SA}}_{\mathrm{it}}=-0.737\times {\mathrm{Size}}_{\mathrm{it}}+0.043\times {\mathrm{Size}}^{2}{}_{\mathrm{it}}-0.04\times {\mathrm{Age}}_{\mathrm{it}} \end{array}$$

where ${\mathrm{Size}}_{\mathrm{it}}$ is the size of firm i in year t and ${\mathrm{Age}}_{\mathrm{it}}$ is the age of firm i in year t. Since SA is generally negative, the larger the absolute value of SA is, the more serious the financing constraint of the enterprise is, so the absolute value of SA is treated.

##### Cash reserves (cash)

The most liquid asset of a company is cash, and operating cash flow shows how well a company can generate cash. This study uses the ratio of net operating cash flow to an organization’s total assets to gauge its cash reserves, and to mitigate possible heteroskedasticity problems, the resulting ratio is treated by adding 1 and taking the natural logarithm (lnCash). It does so by drawing on prior research (Al-Hadi et al., 2020).

#### Control variables

Considering the influence of possible confounding factors, this paper refers to the existing literature and controls for a series of control variables: (1) the level of corporate governance (Bsize), which is determined by the number of boards of directors, because it is generally accepted that businesses with higher levels of corporate governance are more effective in technological innovation (Sapra et al., 2014; Liu et al., 2020); (2) Independence of the board of directors (Bratio), which is measured by the number of independent directors as a percentage of the total number of directors, can increase the market dynamics of the company and thus encourage the company to engage in more R&D and innovation activities (Balsmeier et al., 2017; Nguyen et al., 2020); (3) The maximum shareholder ownership ratio (Sratio), which is considered that a moderate shareholding ratio will stimulate a convergence of interests and thus promote R&D innovation, while too high a shareholding ratio will have a management defense effect and inhibit technological innovation (Mengli and Yongming, 2020); (4) Enterprise development prospects (Future), it is generally believed that more promising companies are more willing to conduct innovative R&D. The growth rate of revenue is used to measure the development capability and prospect of the company (Aguilera-Caracuel and Ortiz-de-Mandojana, 2013; Xie et al., 2022); (5) Firm size (lnAsset), the study concluded that the larger the firm is, the higher its innovation success rate will be, using the logarithm of total assets at year-end to measure firm size (Daksa et al., 2018; Liu et al., 2021); (6) Corporate debt (Lev), which makes it more difficult to carry out corporate innovation activities when a company is in a poor financial position, using the ratio of total debt to total assets to measure a company’s indebtedness (Iqbal et al., 2020); (7) The maturity of the company (Age), research shows that longer established companies have a stronger sense of innovation, and the age of the company is chosen to measure the maturity of the company (Bianchini et al., 2018; Nguyen et al., 2020); (8) Corporate profitability (Share), research shows that the more profitable companies have a competitive advantage in innovation, using earnings per share to measure corporate profitability (Nguyen et al., 2020). Descriptive statistics for each variable are shown in Table 2. From Table 2, the minimum value of lnGInno is 0, the maximum value is 6.811, and the standard deviation is 0.756, indicating that heavy polluting enterprises have uneven attention and commitment to green innovation. The mean value of lnGInnoQ is 0.104 and the variance is 0.271, indicating that overall, the number of invention-based green patent applications of heavy polluting enterprises accounts for a relatively low percentage of green patent applications, which means that the green innovation quality of heavy polluting enterprises is still at a relatively low level. lnEID has a minimum value of 0, a maximum value of 3.996, and a standard deviation of 0.916, indicating that there are differences in the quality of environmental information disclosure by enterprises, and the standard deviation of lnEIDH is 1.103. The standard deviation of lnEIDS is 0.569, implying that the variation of enterprises’ disclosure of hard indicators is more obvious compared to soft indicators. For the control variables, the data on the size of the board of directors, the percentage of independent directors, and the maximum shareholding ratio of the firms are consistent with the actual situation of the heavily polluting listed firms and the statistical results of the existing literature.

**Table 2:** Descriptive statistics.

Variables	Obs	Mean	SD	Min	Max
lnGInno	6,986	0.366	0.756	0	6.811
lnGInnoQ	6,986	0.104	0.271	0	3.575
lnEID	6,986	1.875	0.916	0	3.996
lnEIDH	6,986	1.248	1.103	0	3.616
lnEIDS	6,986	1.355	0.569	0	3.011
SA	6,986	3.843	0.282	1.497	6.541
lnCash	6,986	0.028	0.093	−1.339	1.24
Bsize	6,986	9.901	2.418	0.956	21
Bratio	6,986	0.369	0.061	0.11	0.767
Sratio	6,986	0.621	0.361	−0.004	2.259
Future	6,986	0.156	0.547	−2.944	4.85
lnAsset	6,986	4.133	1.442	−0.795	8.385
Lev	6,986	0.531	0.238	−1.132	1.598
Age	6,986	19.195	5.411	6	43
Share	6,986	0.465	0.614	−1.532	5.425

## Results and discussion

### Benchmark regression

The benchmark regression results from this study are shown in Table 3. The effects of improving the EID quality of high-polluting enterprises on the quantity of green patent applications made by those enterprises are shown in Columns (1) and (2). By comparing Columns (1) and (2), it can be seen that even after several control variables have been added, the effect of improving the EID quality on the quantity of green patent applications made by high-polluting enterprises is still significant at the 1% level, despite its value declining. In particular, for every 1% improvement in the quality of the EID of high-polluting enterprises, the quantity of green patent applications by enterprises will increase by 0.073%; this proves that increasing the quality of the EID of high-polluting enterprises can significantly boost the level of green innovation within enterprises, which is consistent with the conclusions of (Hong et al., 2020). This study also examines how various EID forms affect corporate green innovation. Increasing the quality of corporate EIDH has a numerically more significant promotion effect on the level of corporate green innovation, as can be seen from columns (3) and (4) while increasing the quality of corporate EIDS also has a considerable promotion effect on corporate green innovation. The impact of increasing the EID quality of high-polluting enterprises on the quality of green innovation in enterprises is seen in columns (5) through (7). From column (5), it can be deduced that the proportion of green invention-type patents in enterprises can be significantly increased by improving the EID quality of high-polluting enterprises. For every 1% improvement in EID quality, the proportion of green invention-type patents will rise by 0.024%, that is, high-polluting enterprises. The advancement of green innovation quality of firms can be considerably aided by enhancing the EID quality of enterprises. Columns (6) and (7) show the effects of increasing the quality of EIDH and the quality of EIDS on the quality of green innovation in high-polluting firms, respectively. It is clear that firms have a significant contribution to the quality of green innovation regardless of whether they increase the quality of EIDH or the quality of EIDS, and the contribution of EIDH quality to the quality of green innovation in firms is more outstanding, which is consistent with the existing lite (Johnstone et al., 2017). Compared with soft indicators such as environmental protection philosophy and environmental protection objectives, the public is more concerned about the disclosure of complex indicators such as environmental liabilities and environmental performance disclosed by enterprises and believes that enterprises willing to disclose hard indicators are more responsible and willing to assume their social responsibilities, i.e., disclosure of hard indicators can better help enterprises gain a stamp of legitimacy and enhance their green innovation level. As the main source of pollution, heavily polluting enterprises are the key monitoring objects of the government and the society. In order to highlight their environmental legitimacy, heavily polluting enterprises must continuously improve the quality of their environmental information disclosure, that is, they must not only declare their environmental protection philosophy to the society, but also announce their annual pollutant emissions and the measures taken to cure pollution to the public (Wang et al., 2022). In this context, enterprises must increase their green innovation efforts and improve the quality of green innovation in order to effectively improve their environmental performance, thereby meeting the expectations of the government and the public and ensuring the legitimacy of their own existence, verifying hypothesis 1.

**Table 3:** Benchmark regression.

	(1)	(2)	(3)	(4)	(5)	(6)	(7)
Variables	lnGInno	lnGInno	lnGInno	lnGInno	lnGInnoQ	lnGInnoQ	lnGInnoQ
lnEID	0.219***	0.073**			0.024***		
	(0.044)	(0.028)			(0.007)		
lnEIDH			0.147**			0.046***	
			(0.054)			(0.012)	
lnEIDS				0.043**			0.014***
				(0.020)			(0.004)
Bsize		0.010	0.010	0.011	−0.001	−0.001	−0.001
		(0.009)	(0.010)	(0.009)	(0.002)	(0.002)	(0.002)
Bratio		0.275	0.273	0.265	0.117*	0.116*	0.114*
		(0.284)	(0.286)	(0.284)	(0.064)	(0.065)	(0.064)
Sratio		0.055	0.059	0.057	−0.024	−0.022	−0.023
		(0.079)	(0.080)	(0.079)	(0.031)	(0.031)	(0.031)
Future		−0.047***	−0.045**	−0.050***	−0.005	−0.004	−0.006
		(0.016)	(0.017)	(0.017)	(0.005)	(0.005)	(0.005)
lnAsset		0.228***	0.223***	0.234***	0.043***	0.042***	0.045***
		(0.034)	(0.035)	(0.034)	(0.005)	(0.006)	(0.005)
Lev		−0.010	−0.003	−0.019	−0.003	−0.002	−0.007
		(0.117)	(0.112)	(0.118)	(0.032)	(0.031)	(0.033)
Age		−0.011*	−0.010*	−0.011*	−0.004**	−0.004**	−0.004**
		(0.005)	(0.006)	(0.006)	(0.001)	(0.001)	(0.001)
Share		−0.051*	−0.053*	−0.050	−0.002	−0.002	−0.002
		(0.029)	(0.028)	(0.029)	(0.007)	(0.007)	(0.007)
Constant	0.047	−0.621***	−0.672***	−0.555**	−0.058	−0.073	−0.036
	(0.082)	(0.199)	(0.197)	(0.198)	(0.047)	(0.048)	(0.049)
Year	YES	YES	YES	YES	YES	YES	YES
Industry	YES	YES	YES	YES	YES	YES	YES
Observations	6,986	6,986	6,986	6,986	6,986	6,986	6,986
R^2^	0.183	0.284	0.286	0.282	0.118	0.120	0.117

*, ** and **** represent the significance levels of 10, 5 and 1%, respectively, and heteroskedasticity robust standard errors of the estimated coefficients are in parentheses and adjusted for clustering at the industry level.

### Robust analysis

To verify the robustness of the benchmark regression results, a series of methods were used to test the findings of the benchmark regression (Table 4). First, to mitigate possible endogeneity problems, this paper uses a two-stage least squares (2SLS) approach to validate the results of the benchmark regression. Referring to Bebe Shi et al. (2019), this paper uses the number of types of newspapers in each prefecture-level city as an instrumental variable for environmental information disclosure quality, and further, since the data of the selected instrumental variable are in cross-sectional form, this paper refers to Nunn and Qian (2014), where the mean value of environmental information disclosure quality in each industry in the previous year (related to the time trend) and the number of types of newspapers in each city (related to individual characteristics) as an interaction term for the quality of environmental information disclosure as an instrumental variable. On the one hand, newspapers serve as an important channel for local officials to understand people’s demands, and when environmental issues are found to be the core issues reported in newspapers, local officials are likely to ask firms to improve their environmental information disclosure quality. The number of types of newspapers in a city reflects the local ability to disclose information, and the more types of newspapers, the more likely local firms are to improve their environmental information disclosure quality. On the other hand, the level of green innovation of firms cannot influence the number of types of local newspapers and the mean of environmental information disclosure quality by industry in the previous year (Guan et al., 2020; Shao et al., 2021); therefore, the interaction term of the number of types of newspapers and the mean of environmental information disclosure quality by industry in the previous year satisfies the hypothesis of the instrumental variable. Column (1) reports the estimation results of 2SLS using instrumental variables. From the one-stage regression results, the instrumental variables are significantly positively related to the quality of environmental information disclosure at the 1% statistical level, and the value of the C-D Wald F-statistic is 287.089, which is greater than the critical value at 10% bias (16.38), indicating that there is no weak instrumental variable problem. Column (2) adds both environmental information disclosure quality and instrumental variables, at which time the coefficient of instrumental variables is still positive but no longer statistically significant, further proving that the instrumental variables in this paper can better satisfy the exogeneity hypothesis. From column (1), we can see that after alleviating the endogeneity problem in the model, the improvement of environmental information disclosure quality of heavy polluting enterprises can still significantly promote the improvement of green innovation level of enterprises, which indicates that the results of the baseline regression in this paper are robust and credible. Second, this paper further controls for higher-order fixed effects to prevent potential omitted variables, controls the interaction term between industry and year (column 3) to exclude the influence of dynamic industry characteristics like industry boom and industrial policy, controls the interaction term between province and year (column 4) to exclude the influence of regional economic development, and controls both the interaction term between industry and year and province and year in column 5. The regression results are significant at the 1% level, and the values are the same as those of the benchmark regression, indicating that there is no serious omitted variable problem in the model setting and verifying the robustness of the benchmark regression results. Finally, this paper replaces the number of green patent applications with the number of green patent citations (lnGInnoC) as a proxy variable for firms’ green innovation level. The number of green patent citations of high-polluting enterprises can reflect the green innovation quality of enterprises because it is commonly accepted that the more a patent is cited by later patents, the more significant its influence, and worth. The regression results are displayed in column 6. It has been discovered that increasing the EID quality of heavily polluting enterprises can significantly raise their green patent citations, i.e., raise enterprises’ green innovation level. This finding validates hypothesis 1 and shows that the baseline regression results are robust and credible.

**Table 4:** Robustness test.

	(1)	(2)	(3)	(4)	(5)	(6)
Variables	lnGInno	lnGInno	lnGInno	lnGInno	lnGInno	lnGInnoC
lnEID	0.256***	0.079**	0.077**	0.074**	0.077**	0.006**
	(0.083)	(0.031)	(0.027)	(0.030)	(0.029)	(0.003)
IV		0.021				
		(0.016)				
Bsize	0.005	0.011	0.010	0.011	0.011	0.004
	(0.005)	(0.010)	(0.009)	(0.009)	(0.009)	(0.021)
Bratio	0.453**	0.318	0.285	0.312	0.320	0.000
	(0.185)	(0.305)	(0.281)	(0.278)	(0.275)	(0.004)
Sratio	−0.001	0.038	0.055	0.045	0.046	−0.002
	(0.043)	(0.076)	(0.078)	(0.078)	(0.077)	(0.001)
Future	−0.014	−0.045**	−0.047***	−0.046***	−0.046***	0.003
	(0.015)	(0.016)	(0.016)	(0.016)	(0.016)	(0.002)
lnAsset	0.192***	0.228***	0.225***	0.221***	0.219***	−0.005
	(0.022)	(0.033)	(0.033)	(0.033)	(0.033)	(0.009)
Lev	0.162***	−0.007	−0.010	−0.003	−0.005	−0.001*
	(0.045)	(0.118)	(0.114)	(0.114)	(0.113)	(0.001)
Age	−0.008**	−0.011*	−0.011*	−0.011*	−0.011*	0.006**
	(0.003)	(0.006)	(0.005)	(0.005)	(0.005)	(0.003)
Share	−0.103***	−0.047	−0.054*	−0.049*	−0.052*	0.001
	(0.017)	(0.029)	(0.028)	(0.028)	(0.028)	(0.001)
Constant	−0.573***	−0.693***	−31.794	−0.478**	−32.077	0.004
	(0.300)	(0.219)	(29.435)	(0.192)	(29.231)	(0.015)
c.Year#c.Industry	NO	NO	Yes	NO	Yes	NO
c.Year#c.Province	NO	NO	NO	Yes	Yes	NO
Year	Yes	Yes	Yes	Yes	Yes	Yes
Industry	Yes	Yes	Yes	Yes	Yes	Yes
Observations	6,487	6,487	6,986	6,986	6,986	5489
R^2^	0.142	0.285	0.285	0.288	0.289	0.031
Phase I Regression:						
IV	0.315***					
	(0.039)					
C-D Wald F statistic	287.079					

*, ** and *** represent the significance levels of 10, 5 and 1%, respectively, and heteroskedasticity robust standard errors of the estimated coefficients are in parentheses and adjusted for clustering at the industry level.

### Mediating effect test

To test hypotheses 2 and 3, the mechanism of how high-polluting enterprises’ EID quality affects their green innovation level was examined. Financial constraints can significantly hamper the establishment of innovation projects during the project conceptualization stage, which has been demonstrated to be one of the most significant barriers for businesses to engage in R&D innovation (García-Quevedo et al., 2018). This is because innovation projects consume a significant portion of a company’s resources or have high adjustment costs and uncertainty, and high-polluting enterprises with limited financing may anticipate difficulties obtaining enough money to support their investment in green innovation (Ren et al., 2022a). As a result, they exercise strict control at the beginning of innovation project establishment, which significantly lowers the success rate of innovative project establishment. Column (1) of Table 5 shows that improving the EID quality of heavy polluting enterprises can significantly alleviate the financing constraints faced by enterprises, specifically, for every 1% improvement in the EID quality of enterprises, the absolute value of the SA index of enterprises can be reduced by 2.8%. The combination of columns (1)–(3) shows that improving the EID quality of heavy polluting enterprises can improve the quantity and quality of green innovation by alleviating the financing constraints faced by enterprises, which is the same as the findings of the existing literature and verifies hypothesis 2 (Iqbal et al., 2020). This is because a high-quality EID can signal to investors that enterprises are courageous to take social responsibility and have low environmental risk, alleviate investors’ concerns about the environmental legitimacy of heavy polluting enterprises, and enhance investors’ confidence in future loan and interest recovery, thus alleviating the financing constraints faced by enterprises, which, in turn, adjusts heavy polluters’ expectations of the future financial support they can receive and lowers the approval threshold of heavy polluters for green innovation projects.

**Table 5:** Mediating effect test.

	(1)	(2)	(3)	(4)	(5)	(6)
Variables	SA	lnGInno	lnGInnoQ	lnCash	lnGInno	lnGInnoQ
lnEID	−0.028***	0.074**	0.024***	0.015***	0.072**	0.026***
	(0.008)	(0.030)	(0.007)	(0.003)	(0.029)	(0.007)
SA		−0.992***	−0.105**			
		(0.275)	(0.040)			
lnCash		0.005			0.153*	−0.049*
		(0.008)			(0.078)	(0.029)
Bsize	0.006**	0.159	−0.002	0.001	0.010	−0.001
	(0.002)	(0.270)	(0.002)	(0.001)	(0.009)	(0.002)
Bratio	0.032	0.026	0.105	0.022	0.280	0.117*
	(0.020)	(0.066)	(0.065)	(0.015)	(0.284)	(0.064)
Sratio	−0.008	−0.039**	−0.027	−0.001	0.054	−0.023
	(0.008)	(0.016)	(0.031)	(0.004)	(0.079)	(0.031)
Future	0.010	0.218***	−0.004	0.000	−0.047***	−0.005
	(0.009)	(0.023)	(0.006)	(0.002)	(0.016)	(0.005)
lnAsset	0.119*	−0.175	0.042***	−0.032	0.228***	0.043***
	(0.063)	(0.108)	(0.005)	(0.031)	(0.034)	(0.005)
Lev	0.131***	0.027***	−0.021	−0.052***	−0.012	−0.005
	(0.047)	(0.009)	(0.034)	(0.017)	(0.117)	(0.033)
Age	−0.068***	−0.047	0.000	0.001	−0.011*	−0.004**
	(0.023)	(0.027)	(0.002)	(0.001)	(0.005)	(0.001)
Share	−0.037***	0.005	−0.001	−0.001*	−0.052*	−0.001
	(0.002)	(0.008)	(0.007)	(0.000)	(0.030)	(0.007)
Constant	−3.357***	2.721***	0.295*	0.030	−0.619***	0.077***
	(0.051)	(0.917)	(0.147)	(0.023)	(0.196)	(0.023)
Year	Yes	Yes	Yes	Yes	Yes	Yes
Industry	Yes	Yes	Yes	Yes	Yes	Yes
Observations	6,986	6,986	6,986	6,986	6,986	6,986
R^2^	0.445	0.320	0.122	0.083	0.284	0.118

*, ** and **** represent the significance levels of 10, 5 and 1%, respectively, and heteroskedasticity robust standard errors of the estimated coefficients are in parentheses and adjusted for clustering at the industry level.

Innovation projects have a lengthy and dangerous development cycle, and once they are established, they confine a portion of the company’s resources to use exclusively for the most recent technological innovation and cannot be put to other uses (Argilés-Bosch et al., 2016). A tight capital chain makes it impossible to ensure the project’s smooth progress and increases the unpredictability of the firm’s future status. However, the corporation can mitigate this risk by maintaining cash flow (Al-Hadi et al., 2020). The correlation between the EID of high-polluting enterprises and the proportion of operating cash flow generated by enterprises is seen in columns (4). It has been discovered that increasing the quality of EID for high-polluting enterprises can significantly increase the share of operating cash flow in fixed assets. The value increases by 0.015% for every 1% increase in the quality of EID for enterprises, meaning that increasing the quality of EID for high-polluting enterprises can significantly increase the cash reserves of enterprises. Combining columns (4)–(6), it can be seen that improving the quality of EID of heavy polluting enterprises can promote the quantity and quality of green innovation by increasing the cash reserves of enterprises, which verifies hypothesis 3 and is the same as the conclusion of existing literature (Al-Hadi et al., 2020). High-quality EID can meet the demands of external stakeholders, such as government and society, for heavy polluting enterprises to protect the environment, which makes the connection between enterprises and external stakeholders closer, thus gaining certain competitive advantages, improving the cash flow reserve of heavy polluting enterprises, and then compensating for the shortage of funds encountered by enterprises in the R&D process, and improving the R&D efficiency and R&D success rate of green innovation.

### Heterogeneous analysis

To further verify the robustness of the regression results, this paper examines the heterogeneous effects of the quality of EID of high-polluting enterprises on corporate green innovation (Table 6 and Table 7). First, alternative ownership structures were explored to determine how the EID of high-polluting enterprises affected corporate green innovation (Table 6). By dividing the existing high-polluting enterprises into state-owned enterprises (SOEs) and non-state-owned enterprises (non-SOEs) according to their ownership, it can be obtained from columns (1) and (2) that the improvement in the quality of EID of both SOEs (column 1) and non-SOEs (column 2) significantly promotes the increase in the number of green patent applications. This promotion effect is more evident in non-SOEs, and for every 1% increase in EID quality of high-polluting enterprises, the number of green patent applications of non-SOEs increases by 0.082%, while that of SOEs only increases by 0.063%. As can be seen from columns (3) and (4), state-owned high-polluting enterprises and non-state-owned enterprises will improve the quality of their green patent applications, and this improvement effect is more pronounced for SOEs as compared to non-SOEs. In conclusion, state-owned and non-state-owned high-polluting enterprises can significantly increase their level of green innovation by improving the quality of EID. For non-SOEs, this improvement effect is more evident in the rise of corporate green patent applications, and for SOEs, this improvement effect is more evident in the rise of the quality of EID, in line with (Bortolotti et al., 2022). This may be because non-state-owned high-polluting enterprises face more severe financial constraints than SOEs. That increasing EID quality is more beneficial to easing those financial constraints and providing corresponding financial support for non-SOEs to invest in R&D, while the R&D departments and R&D investment of SOEs are relatively stable, and the number of their green patent applications will not change drastically due to the increase in EID quality. However, it will promote the improvement of their green patent application quality.

**Table 6:** Heterogeneity of firm ownership structure and firm size.

	(1)	(2)	(3)	(4)	(5)	(6)	(7)	(8)
	SOEs	non-SOEs	SOEs	non-SOEs	Large	SMEs	Large	SMEs
Variables	lnGInno	lnGInno	lnGInnoQ	lnGInnoQ	lnGInno	lnGInno	lnGInnoQ	lnGInnoQ
lnEID	0.063**	0.082*	0.042***	0.020***	0.101*	0.044*	0.027**	0.021**
	(0.026)	(0.043)	(0.012)	(0.007)	(0.051)	(0.022)	(0.011)	(0.008)
Bsize	0.011	−0.004	−0.001	−0.001	0.022	−0.006	−0.001	−0.001
	(0.010)	(0.011)	(0.002)	(0.002)	(0.013)	(0.007)	(0.003)	(0.003)
Bratio	0.431	−0.160	0.102	0.154	0.455	0.191	0.218**	0.024
	(0.397)	(0.572)	(0.072)	(0.110)	(0.580)	(0.253)	(0.103)	(0.080)
Sratio	0.014	0.080	−0.008	−0.109**	0.218*	−0.124	0.023	−0.070*
	(0.091)	(0.162)	(0.038)	(0.042)	(0.120)	(0.099)	(0.050)	(0.039)
Future	−0.050**	−0.018	−0.005	−0.008	−0.096***	−0.008	0.001	−0.012*
	(0.019)	(0.026)	(0.007)	(0.012)	(0.028)	(0.016)	(0.011)	(0.006)
lnAsset	0.268***	0.070**	0.051***	0.013**	0.286***	0.094***	0.056***	0.027***
	(0.042)	(0.031)	(0.006)	(0.006)	(0.063)	(0.016)	(0.009)	(0.006)
Lev	−0.008	0.016	−0.003	−0.010	−0.192	−0.028	−0.027	0.011
	(0.098)	(0.178)	(0.039)	(0.032)	(0.207)	(0.088)	(0.043)	(0.035)
Age	−0.004	−0.016*	−0.003**	−0.002	−0.021	−0.010*	−0.004	−0.005
	(0.004)	(0.009)	(0.002)	(0.003)	(0.013)	(0.005)	(0.003)	(0.003)
Share	−0.068**	0.069	−0.003	0.020	−0.060	0.023	−0.001	0.004
	(0.031)	(0.066)	(0.008)	(0.026)	(0.047)	(0.034)	(0.011)	(0.014)
Constant	−0.913***	0.255	−0.094	0.001	−0.929**	0.083	−0.187**	0.077
	(0.235)	(0.309)	(0.063)	(0.085)	(0.368)	(0.241)	(0.067)	(0.110)
Year	Yes	Yes	Yes	Yes	Yes	Yes	Yes	Yes
Industry	Yes	Yes	Yes	Yes	Yes	Yes	Yes	Yes
Observations	5,516	1,470	5,516	1,470	3,486	3,500	3,486	3,500
R^2^	0.329	0.237	0.143	0.083	0.298	0.121	0.140	0.091

*, ** and **** represent the significance levels of 10, 5 and 1%, respectively, and heteroskedasticity robust standard errors of the estimated coefficients are in parentheses and adjusted for clustering at the industry level.

**Table 7:** Heterogeneity in the geographical location of enterprises.

	(1)	(2)	(3)	(4)	(5)	(6)
	Estern	Middle	Western	Estern	Middle	Western
Variables	lnGInno	lnGInno	lnGInno	lnGInnoQ	lnGInnoQ	lnGInnoQ
lnEID	0.172***	0.072*	0.026	0.051***	0.051*	0.012
	(0.063)	(0.041)	(0.036)	(0.018)	(0.028)	(0.013)
Bsize	0.003	0.020	0.006	−0.003	0.010*	−0.007**
	(0.013)	(0.015)	(0.016)	(0.003)	(0.005)	(0.003)
Bratio	0.358	0.441	−0.250	0.225*	−0.057	0.106
	(0.435)	(0.587)	(0.396)	(0.124)	(0.141)	(0.147)
Sratio	0.067	0.012	0.134	−0.064**	0.043	0.012
	(0.130)	(0.116)	(0.129)	(0.030)	(0.062)	(0.047)
Future	−0.074*	−0.074**	0.008	−0.013	0.011	−0.007
	(0.041)	(0.034)	(0.032)	(0.008)	(0.016)	(0.010)
lnAsset	0.262***	0.154***	0.164***	0.053***	0.026**	0.033***
	(0.034)	(0.040)	(0.039)	(0.007)	(0.012)	(0.012)
Lev	−0.092	0.110	0.128	−0.020	0.042	0.004
	(0.164)	(0.144)	(0.100)	(0.033)	(0.042)	(0.037)
Age	−0.020*	−0.022	−0.002	−0.004*	−0.008	−0.005
	(0.011)	(0.015)	(0.011)	(0.002)	(0.005)	(0.003)
Share	−0.065	0.050	−0.087**	0.001	0.005	−0.002
	(0.052)	(0.054)	(0.040)	(0.014)	(0.020)	(0.017)
Constant	−0.528**	−0.366	−0.421	−0.102	−0.052	0.067
	(0.266)	(0.433)	(0.330)	(0.076)	(0.092)	(0.119)
Year	Yes	Yes	Yes	Yes	Yes	Yes
Industry	Yes	Yes	Yes	Yes	Yes	Yes
Observations	3,549	1,747	1,690	3,549	1,747	1,690
R^2^	0.335	0.321	0.289	0.149	0.126	0.178

*, ** and **** represent the significance levels of 10, 5 and 1%, respectively, and heteroskedasticity robust standard errors of the estimated coefficients are in parentheses and adjusted for clustering at the industry level.

Second, the relationship between firm size and the extent of green innovation in high-polluting enterprises was investigated (Table 6). According to total year-end assets, firms were separated into categories based on size. If their total year-end assets exceeded the 75% quantile of all firms’ total year-end assets, they were classified as large enterprises (Large), otherwise as small and medium-sized enterprises (SMEs). The effect of increasing the EID quality of large, high-polluting enterprises on the quantity of their green patent applications is shown in columns (5) and (6). Increasing the EID quality of both large and SMEs can significantly increase the number of green patent applications of the businesses, but this promotion effect is more substantial for large businesses. Green patent applications from large, high-polluting enterprises often increase by 0.1% for every 1% EID quality, whereas those from SMEs typically increase by 0.044%. Columns (7) and (8) show the effects of increasing the EID quality of various-sized enterprises on the quality of green patent applications, demonstrating that increasing the EID quality of large and high-polluting enterprises is more likely to increase the quality of their green patent applications than that of SMEs. This is in line with the results of Ding et al. (2022) and could be explained by the fact that an enterprise’s size affects how effectively it innovates and how often it succeeds, whereas SMEs tend to be less willing to innovate and less successful at it because of resource and expertise limitations.

Finally, the effect of EID quality on high-polluting enterprises’ green innovation under the circumstances of various geographic locations was examined (Table 7). The regressions were carried out separately for three groups of high-polluting enterprises according to the geographical locations of the enterprises, namely, eastern (including 11 provinces and cities on the northeast and east coast), central (including eight provinces), and western (including 12 provinces, cities, and autonomous regions). In Table 7, columns (1) to (3) show the correlation between the quantity of green patent applications filed in various regions and the quality of the EID of high-polluting enterprises, and columns (4) to (6) show the correlation between the quantity of green patent applications filed in various regions and the quality of the EID of high-polluting enterprises. It can be inferred from columns (1) through (3) that while the promotion effect has not been demonstrated in the west, the enhancement of EID quality at high-polluting enterprises in the east and central regions can significantly spur the growth of their green patent applications. The growth of the high-polluting enterprises in the east can encourage the growth of their green patent applications more than those in the middle, as seen by comparing columns (1) and (2). From columns (4) to (6), it is clear that the quality of green patent applications can be significantly improved by improving the EID quality of the high-polluting enterprises located in the eastern and central parts of China. This improvement effect is more pronounced for the enterprises located in the east, whereas the influence of the improvement of EID quality of the high-polluting enterprises located in the west on the quality of green patent applications is less noticeable. It can be concluded that the level of green innovation contributed by high-polluting enterprises decreases from east to west and that the level of green innovation contributed by enterprises in the western region does not significantly increase as the EID quality of high-polluting enterprises increases in this region, which is consistent with the findings of existing literature (Li G. et al., 2022). This may be because the eastern coastal region of China, in comparison to the central and western regions, has a higher level of development and, consequently, a higher level of human capital. It also has the capital and human resource base necessary for green innovation, which can help local businesses improve their green innovation through economic agglomeration and knowledge spillover.

## Conclusion, limitations, and future research directions

Enterprises can provide high-quality environmental information to advance both high-quality economic development and high-level ecological environment conservation. Studying the connection between corporate green innovation and the quality of Environmental information disclosure can increase the importance of EID by enterprises and help them recognize its value, which is very important practice for China to achieve a “win-win” situation of economic development and environmental protection. This study examines the impact of the EID quality of high-polluting enterprises on corporate green innovation by using high-polluting enterprises listed in China from 2008 to 2018 as the research sample. It classifies the EID made by high-polluting enterprises (EIDS and EIDH), calculates the EID quality index of high-polluting enterprises, and studies the influence of the EID quality of high-polluting enterprises on corporate green innovation. This paper uses the high-polluting enterprises listed in China from 2008 to 2021 as the research sample, classifies the environmental information disclosed by high-polluting enterprises (EIDS and EIDH), calculates the EID quality index of high-polluting enterprises, and studies the influence of EID quality of high-polluting enterprises on corporate green innovation.

The results show that improving the quality of EID of heavy polluting enterprises can make the level of green innovation “increase in quantity and improve in quality,” and further breakdown of EID of enterprises shows that both EIDH and EIDS can improve the quantity and quality of green innovation of enterprises. Robustness analysis shows that the above findings are reliable. The mechanism analysis demonstrates that by reducing the financial restrictions, high-polluting enterprises have and boosting their cash reserves, enhancing the quality of their EID can increase the degree of green innovation in enterprises. The encouragement of green innovation by the EID quality of high-polluting enterprises is impacted by differences in ownership structure, enterprise size, and geographic location. Specifically, improving enterprise EID quality is more likely to enhance the number of green patent applications of non-SOEs and the quality of green patent applications of SOEs. Compared with SMEs, improving EID quality of large enterprises can promote the level of green innovation of enterprises. Compared with the central and western regions, the improvement of EID quality of enterprises in the eastern region is more capable of enhancing the green innovation level of high-polluting enterprises in that region, followed by the central region, and the promotion effect of the improvement of EID quality of enterprises in the western region on the green innovation of high-polluting enterprises in that region has not yet appeared.

This report suggests the following policy recommendations based on the findings as mentioned above:

First, to increase the promotion effect of EID on the degree of green innovation, pertinent government departments should further standardize the guidelines and evaluation criteria for EID and improve the quality of EID by enterprises. The depth and breadth of EID for firms should be significantly increased, necessitating that the whole product declaration cycle be covered in time, and the commercial scope conducted by enterprises at home and abroad be included in space.

Second, it should further promote the development of a green financial system, make the quality of EID of enterprises one of the critical reference criteria for whether enterprises can receive green credit, and simultaneously emphasize the significance of environmental protection to the general public, cultivate their attention to environmental protection. As a result, enterprises must disclose environmental information more accurately while easing their financial and cash flow limitations.

Finally, the government must implement specific and targeted measures to encourage the improvement of the green innovation level of relevant enterprises. These measures include vigorously supporting SMEs with policies, increasing their credit supply and removing corresponding financial restrictions, increasing their access to capital, and reducing regulatory burdens.

The paper also has certain limitations that need to be improved in the future. First, the future study can use pertinent institutions’ assessment findings of the EID quality of firms, and this paper manually rates the EID quality of enterprises, which is somewhat subjective. Second, future research can use the entire industry as a sample to examine the impact of EID quality on green innovation in all firms. This study only looked at the effects of enhancing EID quality on corporate green innovation in listed companies with significant pollution. Finally, future studies can examine if increasing businesses’ EID quality will encourage green innovation at the expense of other forms of innovation. This paper only looked at how EID affected corporate green patents, it did not examine if it may crowd out other enterprise patents.

## Data availability statement

The original contributions presented in the study are included in the article/supplementary material, further inquiries can be directed to the corresponding authors.

## Author contributions

LD and XW: conceptualization and methodology. XW, GJ, and SD: resources. XW and JP: formal analysis and writing—original draft preparation. LD, XW, and JP: writing— review and editing. All authors contributed to the article and approved the submitted version.

## Funding

This work was supported by the National Social Science Funds of China under Grant 17BJL058.

## Conflict of interest

The authors declare that the research was conducted in the absence of any commercial or financial relationships that could be construed as a potential conflict of interest.

## Publisher’s note

All claims expressed in this article are solely those of the authors and do not necessarily represent those of their affiliated organizations, or those of the publisher, the editors and the reviewers. Any product that may be evaluated in this article, or claim that may be made by its manufacturer, is not guaranteed or endorsed by the publisher.

## Footnotes

^1^Sixteen highly polluting sectors, respectively, thermal power, iron and steel, cement, electrolytic aluminum, coal, metallurgy, chemicals, petrochemicals, building materials, paper, brewing, pharmaceuticals, fermentation, textiles, tannery and mining.
